# Mitigation of sepsis-induced inflammatory responses and organ injury through targeting Wnt/β-catenin signaling

**DOI:** 10.1038/s41598-017-08711-6

**Published:** 2017-08-23

**Authors:** Archna Sharma, Weng-Lang Yang, Mahendar Ochani, Ping Wang

**Affiliations:** 1 Center for Immunology and Inflammation, The Feinstein Institute for Medical Research, Manhasset, NY 11030 USA; 2 Department of Surgery, Hofstra Northwell School of Medicine, Manhasset, NY 11030 USA

## Abstract

The Wnt/β-catenin pathway has been involved in regulating inflammation in various infectious and inflammatory diseases. Sepsis is a life-threatening condition caused by dysregulated inflammatory response to infection with no effective therapy available. Recently elevated Wnt/β-catenin signaling has been detected in sepsis. However, its contribution to sepsis-associated inflammatory response remains to be explored. In this study, we show that inhibition of Wnt/β-catenin signaling reduces inflammation and mitigates sepsis-induced organ injury. Using *in vitro* LPS-stimulated RAW264.7 macrophages, we demonstrate that a small-molecule inhibitor of β-catenin responsive transcription, iCRT3, significantly reduces the LPS-induced Wnt/β-catenin activity and also inhibits TNF-α production and IκB degradation in a dose-dependent manner. Intraperitoneal administration of iCRT3 to C57BL/6 mice, subjected to cecal ligation and puncture-induced sepsis, decreases the plasma levels of proinflammatory cytokines and organ injury markers in a dose-dependent manner. The histological integrity of the lungs is improved with iCRT3 treatment, along with reduced lung collagen deposition and apoptosis. In addition, iCRT3 treatment also decreases the expression of the cytokines, neutrophil chemoattractants, as well as the MPO activity in the lungs of septic mice. Based on these findings we conclude that targeting the Wnt/β-Catenin pathway may provide a potential therapeutic approach for treatment of sepsis.

## Introduction

Sepsis is now defined as a clinical syndrome due to dysregulated systemic immune response to infection that causes multiple organ failure and could be life-threatening^1^. Sepsis is associated with high morbidity and mortality and is arguably one of the leading causes of preventable death in the world today^2–5^. In spite of the remarkable efforts and money spent with the objective of developing treatments, there is still no effective drug available, other than antibiotics, vasopressors and supportive care^6, 7^. The pathophysiology of sepsis is still poorly understood, even after extensive basic research and clinical studies. Early phase of sepsis is characterized by a complex and dynamic systemic host response manifested by an array of pro-inflammatory mediators accompanied by numerous counter-regulatory mechanisms causing large scale organ damage and death^8, 9^. The dysregulated inflammatory response in sepsis is a result of many diverse and cross-regulated pathways which gets altered^10^. Certainly, understanding the diverse signaling pathways activated and cross regulated during sepsis will impact the search for new therapeutic targets and agents with the compelling need to treat sepsis.

The canonical Wnt pathway is well characterized and involves β-catenin and members of T-cell factor (TCF)/lymphoid enhancer-binding factor (LEF) family of transcription factors (TCF/LEF). Activation of the Wnt/β-catenin pathway via Wnt ligands prevents the proteasomal degradation of β-catenin by inhibiting the glycogen synthase kinase 3 β (GSK3β) phosphorylation activity, resulting in accumulation and translocation of β-catenin to the nucleus where it drives the expression of TCF/LEF-dependent genes^11, 12^. Interestingly, Wnt signaling, classically regarded as the pathway involved in the control of cell proliferation, migration, and differentiation in embryonic development, has recently been involved in immunoregulatory mechanisms in various infectious and inflammatory diseases^13, 14^.

The canonical Wnt signaling was shown to be activated by TLR4-ligand lipopolysaccharide (LPS) in monocytes and macrophages, *via* a mechanism dependent on PI3K/AKT and Erk pathways, indicating towards its contribution to inflammation^15, 16^. Like TLR4, other TLRs such as TLR2, TLR3, TLR5, and TLR9 are also known to activate or regulate β-catenin signaling in a pathogen or cell type-specific manner^14^. However, only limited evidence is available for a role of canonical Wnt/β-catenin signaling in sepsis. Activation of Wnt signaling has been reported in the lungs during the early stage of sepsis^17, 18^. Interestingly, Wnt/β-catenin signaling is involved in the progression of inflammatory lung diseases including asthma^19, 20^, emphysema^21^, and pulmonary fibrosis^22, 23^. A recent study showed that Wnt inhibitors suppress LPS-induced inflammatory responses, hinting that a therapeutic strategy designed to attenuate Wnt/β-catenin signaling has the potential to prevent sepsis-induced inflammation^24^.

In the present study, we used iCRT3 [chemical name: 2-(((2-(4-Ethylphenyl)-5-methyl-1,3-oxazol-4-yl)methyl)sulfanyl)-N-(2-phenylethyl)acetamide], a small cell-permeable oxazole compound, which acts as a selective inhibitor of the Wnt pathway by blocking the interaction of β-catenin-TCF via direct binding to β-catenin^25^. The effect of iCRT3 on Wnt/β-catenin signaling and proinflammatory activity in LPS-stimulated macrophages was first demonstrated by assessing the inhibition of TCF reporter activity, cytokine production and IκB degradation. We then examined the effect of treatment with iCRT3 on inflammation and organ injury in mice with sepsis induced by cecal ligation and puncture (CLP), a physiologically relevant model. This approach not only further elaborated the role of β-catenin-TCF mediated Wnt signaling in regulating sepsis-induced inflammation and organ injury but also evaluated the potential of using Wnt/β-catenin signaling-inhibitors as a therapeutic strategy for treating sepsis-induced lung damage.

## Results

### iCRT3 inhibits cytokine production in LPS-stimulated macrophages

Release of a cascade of proinflammatory cytokines from macrophages is associated with the “cytokine storm” during sepsis. We first determined the effectiveness of iCRT3 in altering Wnt/β-catenin signaling in macrophages in response to LPS. The murine alveolar RAW264.7 macrophage cells were co-transfected with β-catenin/TCF response reporter TOP-TK-Luc or its control FOP-TK-Luc with *Renilla* luciferase reporter RL-TK. The tranfected cells were pre-treated with iCRT3 followed by LPS stimulation. Dual-luciferase assay demonstrated no detectable Wnt/β-catenin signaling activity as baseline in the naïve RAW264.7 cells. Wnt/β-catenin signaling reported by TOP-TK was increased by 3.2-fold in the cells treated with LPS, whereas FOP-TK showed no activation as expected (Fig. 1A). Treatment with iCRT3 significantly reduced the LPS-induced TOP-TK reporter activity by 32% (Fig. 1A).

**Figure 1:** Effect of iCRT3 on Wnt/β-catenin activation and TNF-α production in LPS-stimulated macrophages. Cultured RAW 264.7 cells were pre-treated with iCRT3 at the indicated concentration for 50 min and then stimulated with LPS (1 ng/ml). **(A)** Before treatment, RAW264.7 macrophage cells were co-transfected with β-catenin/TCF response reporter TOP-TK-Luc or its control FOP-TK-Luc and an internal control pRL-TK. Luciferase activity was measured after 24 h LPS stimulation and expressed as the relative fold change compared to the untreated. **(B)** Supernatants from cultured RAW 264.7 cells were subjected to ELISA for measurement of TNF-α level after 4 h LPS stimulation. **(C)** Cell viability of RAW 264.7 cells was determined by MTS assay with viability of untreated cells considered to be 100%. **(D)** Western blotting against IκB and actin using total cell lysate after 15 min LPS stimulation. The image shown is representative of three independent experiments with bar graph from densitometric analysis of blots. Data were expressed as mean ± SEM obtained from two independent experiments (n = 4 per group). *P < 0.05 versus vehicle and ^#^ *P* < 0.05 versus LPS alone.

Next, we measured the TNF-α levels in the supernatants from RAW 264.7 cells pretreated with iCRT3 and stimulated with LPS. After 4 h-LPS stimulation, the TNF-α levels in cultured RAW264.7 cells reached 6.8 ng/ml, while treatment with iCRT3 at doses of 12.5, 25, 50, and 75 μM decreased TNF-α levels by 14.7%, 18.5%, 44.9% and 61.3%, respectively (Fig. 1B). We also examined the viability of RAW 264.7 cells and observed no adverse effects of iCRT3 on cell viability (Fig. 1C). The levels of IκB, an NF-κB inhibitor, in RAW 264.7 cells were decreased by one-third in the total cell extract, after LPS stimulation (Fig. 1D). With iCRT3 treatment, IκB levels were increased in a dose-dependent manner compared to the vehicle (Fig. 1D). These results indicate that iCRT3 inhibited Wnt/β-catenin signaling as well as the pro-inflammatory cytokine production from macrophages potentially via NF-κB-mediated pathway.

### iCRT3 treatment reduces the systemic inflammation and organ injury in sepsis

After demonstrating that iCRT3 inhibits pro-inflammatory cytokine production *in vitro*, we then administered iCRT3 to mice that underwent sepsis-induction by CLP and examined the plasma levels of pro-inflammatory cytokines. As increased plasma IL-6 levels have been correlated with the severity of sepsis^26^, at 20 h after CLP, we found IL-6 plasma levels were significantly increased by 10.7-fold in the vehicle group, compared to the sham group (Fig. 2A). However, the IL-6 levels in the 10 mg/kg iCRT3 treatment group were 82.9% lower than those in the vehicle group (Fig. 2A). Plasma levels of another proinflammatory cytokine TNF-α were also 522-fold higher in the vehicle group than the sham group and were decreased by 32.9% and 53.9% with respective iCRT3 treatment doses (Fig. 2B). IL-1β levels were undetectable in the sham but reached 371 pg/ml in septic mice and were down by 30.2% and 53.2%, respectively, with 5 and 10 mg/kg iCRT3 (Fig. 2C).

**Figure 2:** Effect of iCRT3 administration on systemic cytokine levels after CLP. Male C57BL/6 mice were sham-operated or subjected to CLP with vehicle (5% DMSO in normal saline) or iCRT3 (5 mg/kg and 10 mg/kg body weight) treatment at 5 h after CLP. Blood samples were collected at 20 h after CLP to measure **(A)** IL-6, **(B)** TNF-α, and **(C)** IL-1β by using ELISA. Data were expressed as means ± SEM (n = 5–8 mice per group). *P < 0.05 versus sham and ^#^ *P* < 0.05 versus vehicle-treated septic animals.

Excessive levels of circulatory pro-inflammatory cytokines are known to contribute to sepsis-induced remote organ injury. Accordingly, at 20 h after CLP, the plasma levels of broad range organ damage marker AST were significantly increased by 12.5-fold in the vehicle group, compared to the sham group (Fig. 3A). However, with iCRT3 treatment at doses of 5 and 10 mg/kg, AST levels in these septic mice were 15.4% and 44.2% lower, respectively, than those in the vehicle-treated mice (Fig. 3A). The levels of more liver injury-specific marker ALT, in these septic mice were increased by 5.9-fold relative to sham, with iCRT3 treatments bringing them down dose-dependently by 24.8% and 42.9% (Fig. 3B). Similarly, levels of another common tissue damage marker LDH in these septic mice were 10.9-fold higher and were reduced by 27.7% and 56.9%, respectively after 5 and 10 mg/kg iCRT3 treatment (Fig. 3C). Taken together, these results indicated that administration of iCRT3 resulted in the reduction of systemic levels of pro-inflammatory cytokines and organ injury markers in septic mice.

**Figure 3:** Effect of iCRT3 administration on plasma levels of organ injury markers after CLP. Male C57BL/6 mice were sham-operated or subjected to CLP with intraperitoneal injection of vehicle (5% DMSO in normal saline) or iCRT3 (5 mg/kg and 10 mg/kg body weight) at 5 h after CLP. Blood samples were collected at 20 h after CLP to measure **(A)** AST, **(B)** ALT, and **(C)** LDH by using the commercial assay kit. Data were expressed as means ± SEM (n = 5–8 mice per group). *P < 0.05 versus sham and ^#^ *P* < 0.05 versus vehicle-treated septic animals.

### iCRT3 treatment attenuates sepsis-induced lung injury

Considering that acute lung injury is clearly identified as a serious and very frequent complication in sepsis^27^, we examined the histological architecture of lungs at 20 h post-CLP. Substantial morphological changes were observed in the lung tissues of the vehicle-treated group, including alveolar collapse, congestion with edema, hemorrhage, and infiltration of neutrophils, compared to the sham group (Fig. 4A). After treatment with 10 mg/kg iCRT3, lung morphology was improved with much reduced microscopic deterioration, compared to the vehicle group (Fig. 4A). We further quantified the severity of histological lung damage, with vehicle group showing 13.7-fold increase in the injury score compared to the sham group and iCRT3 treatment significantly reducing it by 53.6% (Fig. 4B).

**Figure 4:** Histological analysis of lungs after CLP and iCRT3 treatment. Male C57BL/6 mice were subjected sham operation or CLP with vehicle (5% DMSO in normal saline) or 10 mg/kg body weight iCRT3 injections at 5 h after CLP. The lung tissues were harvested at 20 h after CLP. (**A**,**B**) Sections of lung tissues were stained with H&E and examined under light microscopy. Representative images at original magnification ×200 **(A)** and graph of histological lung injury scores **(B)**, determined as described in Materials and methods are shown. **(C**,**D)** Sections of lung tissues were stained with Masson’s Trichrome and examined under light microscopy. Representative images at original magnification ×200 **(C)** and × 400 **(D)** are shown. Data were expressed as means ± SEM (n = 4 per group). *P < 0.05 versus sham and ^#^ *P* < 0.05 versus vehicle-treated septic animals.

Collagen deposition is an early event during sepsis-induced acute lung injury and excessive collagen deposition in the lungs leads to destruction of lung architecture^28, 29^. So next, we performed the Masson Trichrome staining to examine lung collagen levels (Fig. 4C,D). Collagen was identified in sham lungs only in areas surrounding large vessels and bronchioles (Fig. 4C). However, lungs from septic animals in the vehicle group showed focal areas of collagen deposition in the parenchyma as well as proteinaceous exudate in the intra-alveolar spaces (Fig. 4C,D). After iCRT3 treatment the collagen deposition did not appear as extensive as observed in the vehicle lungs, both in areas surrounding bronchioles as well as in parenchyma (Fig. 4C,D). Our findings suggest that iCRT3 treatment improved CLP-induced lung damage and attenuated collagen deposition in the lungs.

### iCRT3 treatment decreases apoptosis and inflammation in the lungs of septic mice

Apoptotic cell death has been considered an underlying mechanism in acute lung injury. We performed TUNEL assay in the lung tissues to investigate the effect of iCRT3 treatment on lung apoptosis. The number of TUNEL-positive cells in the lung tissues of the vehicle group was distinctly increased compared to the sham groups (Fig. 5A). Interestingly, the number of apoptotic cells in the lung tissues of the iCRT3-treated mice was significantly reduced by 92.7% in comparison with the vehicle group (Fig. 5B).

**Figure 5:** Detection of apoptosis in the lungs of septic mice treated with iCRT3. Male C57BL/6 mice were subjected to sham-operation or CLP with vehicle (5% DMSO in normal saline) or 10 mg/kg body weight iCRT3 injected in the peritoneum at 5 h after CLP. The lung tissues were harvested at 20 h after CLP. Sections of lung tissues were stained with TUNEL and examined under fluorescent microscopy. **(A)** Representative images at original magnification ×200 are shown. **(B)** The numbers of apoptotic cells quantified from the TUNEL staining (averaged over 10 microscopic fields per mouse) are shown. Data were expressed as means ± SEM (n = 4 sections per group). *P < 0.05 versus sham and ^#^ *P* < 0.05 versus vehicle-treated septic animals.

Next, we measured the local expression of proinflammatory cytokines IL-6, TNF-α, and IL-1β, the NF-κB signaling targets, in the lungs. The mRNA levels of these cytokines were markedly elevated after CLP compared to sham (Fig. 6). Treatment with iCRT3 significantly reduced the expression levels of IL-6, TNF-α, and IL-1β by 98.4%, 76.9% and 79.8%, respectively, in comparison with the vehicle group (Fig. 6).

**Figure 6:** Effect of iCRT3 treatment on the expression of cytokines in the lungs after CLP. CLP-operated male C57BL/6 mice were injected with vehicle or iCRT3 (10 mg/kg body weight) at 5 h post-CLP. Sham-operated mice were used as controls. The lung tissues were harvested at 20 h after CLP. The levels of **(A)** IL-6, **(B)** TNF-α, and **(C)** IL-1β mRNA, in the lung tissue homogenates were determined by qPCR. The results of qPCR analysis are normalized with actin as an internal control and are expressed as fold induction compared to the sham group. Data were expressed as means ± SEM (n = 5–8 mice per group). *P < 0.05 versus sham and ^#^ *P* < 0.05 versus vehicle-treated septic animals.

### iCRT3 treatment reduces neutrophil infiltration in the lungs in sepsis

Excessive neutrophil sequestration and activation is a critical factor causing acute lung injury in sepsis^30, 31^. First, we determined the expression of neutrophil attracting chemokines, macrophage inflammatory protein 2 (MIP-2) and keratinocyte-derived chemokine (KC), in the lungs. Similar to cytokines, mRNA levels of both chemokines MIP-2 and KC in the lungs were highly increased after CLP, but strikingly inhibited with iCRT3 treatment by 96.9% and 93.3%, respectively (Fig. 7A,B). To evaluate the neutrophil content in the lungs, we assessed MPO activity as a marker for neutrophil infiltration. In consistence, there was a 10.3-fold increase of the lung MPO activity in the vehicle group compared to the sham group, which was reduced by 69.6% with iCRT3 treatment (Fig. 7C).

**Figure 7:** Effect of iCRT3 treatment on the neutrophil infiltration in the lungs after CLP. The lung tissues from sham, vehicle and 10 mg/kg body weight iCRT3-treated mice were harvested at 20 h after CLP. The levels of **(A)** MIP-2, and **(B)** KC mRNA, in the lung tissue homogenates were determined by qPCR. The results of qPCR analysis are normalized with actin as an internal control and are expressed as fold induction compared to the sham group. **(C)** Lung tissues were homogenized and MPO activity was determined spectrophotometrically. Data were expressed as mean ± SEM (n = 5–8 mice per group). *P < 0.05 versus sham and ^#^ *P* < 0.05 versus vehicle-treated septic animals.

## Discussion

Even after new guidelines and advances in the management and care of sepsis patients, a large number die from the consequent septic shock and organ failure, posing a dire need of innovative approaches to find targets and design therapeutics for sepsis^4^. Undoubtedly, a major contributing factor for causing sepsis-induced organ injury is the excessive systemic and local inflammation. The cause of this immune-dysregulation is the complex interplay of diverse signaling pathways which gets aberrantly activated or suppressed losing their normal regulated functions^10^. The significance of β-catenin signaling involved in regulating inflammation and injury in sepsis has not been addressed.

In this study, we evaluated iCRT3, a small molecule inhibitor of the Wnt pathway which binds to β-catenin interfering with its interaction with TCF^25^, for its effect on inflammatory macrophage activity. We confirmed its inhibitory effect on Wnt/β-catenin signaling via TOP-TK reporter activity and further demonstrated its effect on reducing cytokine production and IκB degradation in RAW264.7 macrophages *in vitro*. We then illustrated, using an *in vivo* CLP-induced sepsis model, that post-treatment with iCRT3 significantly reduces the systemic inflammatory response and attenuates organ damage in septic mice. We also showed that iCRT3 treatment improves the lung tissue integrity with decreased collagen deposition in the lungs. Furthermore, iCRT3 treatment effectively inhibits the local pro-inflammatory cytokine expression and decreases the lung apoptosis. Finally, administration of iCRT3 attenuated expression of neutrophil attracting chemokines and neutrophil infiltration demonstrated by reduced MPO activity in the lungs of iCRT3 treated septic mice. These findings are summarized in Fig. 8.

**Figure 8:** Summary of effects of blocking Wnt/β-catenin signaling in sepsis. Wnt/β-catenin signaling is upregulated in macrophages after LPS stimulation and during sepsis, which then upregulates NF-κB signaling, resulting in increased systemic and local proinflammatory cytokines and chemokines, as well as increased collagen deposition, apoptosis and neutrophil infiltration in the lungs leading to organ injury. Treatment with iCRT3 blocks the Wnt/β-catenin signaling and reverses these changes attenuating sepsis-induced inflammatory responses and organ injury.

LPS has been shown to stimulate cytosolic β-catenin accumulation and signaling required for target gene transcription and cell migration in macrophages^15, 16^. Similar to these findings, LPS stimulated the Wnt/β-catenin signaling in RAW264.7 macrophages. Pre-treatment with iCRT3 resulted in attenuation of Wnt/β-catenin signaling. We further demonstrated that blocking Wnt/β-catenin signaling by iCRT3 resulted in a dose-dependent attenuation of TNF-α production by RAW264.7 macrophages. We did not observe the effect of iCRT3 treatment on macrophage viability, which indicates that the reduction of TNF-α levels by iCRT3 is not due to macrophage death during the assay. The degradation of IκB controls the activation of NF-κB signaling, which is crucial for the macrophage cytokine production^32, 33^. The anti-inflammatory activity of iCRT3 was further demonstrated by inhibition of the LPS- induced IκB degradation by iCRT3 pre-treatment in a dose-dependent fashion. We examined TNF-α and IκB expression levels with regard to NFκB signaling in this study because TNF-α contains NFκB binding site in its promoter^34^. The change of TNF-α expression corresponded to the IκB levels, which implicates the translocation of NFκB to regulate the TNF-α expression.

In support of our findings, β-catenin has been reported to positively regulate NF-κB activity, as well as the expression of inflammatory cytokines in the inflammatory response of LPS-treated bronchial epithelial cells^35^. Furthermore, LGK974, a small molecular inhibitor of the Wnt secretion, suppressed the LPS-induced IκB degradation and NF-κB nuclear translocation as well as the expressions of pro-inflammatory genes in a dose-dependent and β-catenin-mediated manner^24^. However, another study which used small interfering RNA to dissect role of β-catenin in LPS-induced inflammatory response in RAW264.7 macrophages, reported a negative regulation of IL-6 mRNA expression and NF-κB activity^19^. The Wnt-signaling inhibitor iCRT3 used in our study, disrupts interaction of β-catenin with TCF family members specifically inhibiting the downstream β-catenin responsive transcriptional activity, without having any effect on the protein levels of β-catenin^25^. In contrast, the results from the study by Lee *et al*. were based on decreased protein levels of β-catenin^19^. The difference between the experimental conditions as well as the techniques to target Wnt/β-catenin signaling might explain the contrasting results. In addition to the canonical pathway, several other noncanonical Wnt signaling pathways also exist which are β-catenin-independent^36^. Wnt5A is upregulated in sepsis and is reported to be critically involved in inflammatory macrophage signaling via non-canonical Wnt5A/CaMKII pathway^37, 38^. On the contrary, another study reported that Wnt5a induces immune-suppressive macrophages in sepsis^39^. This is not surprising as Wnt signaling is known to prevent or promote inflammation depending on the cellular context, the type of insult, and the cytokine environment^13, 14^.

Based on *in vitro* effectiveness of iCRT3 in inhibiting inflammatory cytokine production from macrophages, we then attempted to administer iCRT3 in CLP-induced sepsis model. The plasma analysis showed that the levels of IL-6, TNF-α, and IL-1β, are significantly reduced dose-dependently with iCRT3 treatment. Interestingly, the synthesis of these proinflammatory cytokines is mediated by the NF-κB signaling^40^. A proinflammatory role of Wnt signaling is well documented^37, 38, 41^. Thus, iCRT3 blocks the downstream events of both Wnt/β-catenin and NF-κB signaling *in vivo* as well. Inflammasome is the mechanism to control IL-1β release, while the expression of pro-IL-1β is controlled by the activation of NFκB. As we demonstrated *in vitro* that iCRT3 effectively inhibited NFκB activation, which may be the major mechanism contributing to the decrease of plasma IL-1β levels. Whether iCRT3 involves in regulating the inflammasome assembly needs to be further explored. Interestingly, GSK-3β inhibition has also been shown to reduce the proinflammatory response in mice and rats after LPS-induced endotoxin shock via attenuation of NFκB signaling^42, 43^. However, GSK-3β inhibition affects many diverse signaling pathways. Whether its attenuation of NFκB signaling is through the activation of Wnt/β-catenin signaling is not clear. Several organ injury markers (AST, ALT and LDH) are also attenuated in septic mice after iCRT3 treatment in a dose-dependent manner. Our results further validate the link between Wnt/β-catenin signaling and hyperinflammation/multiple organ injury in sepsis, with administration of iCRT3 effectively attenuating both.

We examined the lung injury in septic mice, in more detail. CLP induced severe damage in the lung tissues as demonstrated by histologic analysis. After iCRT3 treatment, the structural integrity of the lung was better protected, with statistically significant improvement in lung injury score as judged by histologic examination. Early collagen deposition in rat lungs in CLP and LPS-induced sepsis model has been observed recently and associated with Wnt/β-catenin signaling activation^18, 44^. In accordance with these findings, increased collagen deposition in the lungs of septic mice was also evident in our study. Interestingly, effectiveness of iCRT3 in blocking Wnt/β-catenin pathway and attenuating collagen deposition in the bleomycin-induced fibrotic lung injury model has also been demonstrated previously^23^. These studies further support the approach of targeting Wnt/β-catenin signaling using small molecule inhibitors to control lung injury in sepsis. In addition to lung injury, acute kidney injury is also often observed in the septic patients^45^. Whether iCRT3 treatment can also attenuate kidney injury induced by sepsis needs further investigation.

Of note, the protective effect of blocking Wnt/β-catenin pathway in pulmonary fibrosis via small interfering RNA (siRNA) for β-catenin, was attributed to the inhibition of collagen synthesis, by reducing TGF-β and matrix metaloproteinase-2 expression, with no significant effect on the inflammatory response^46^. However, when Wnt/β-catenin signaling was inhibited in bleomycin-induced lung fibrosis in mice using small molecule inhibitors XAV939 (works via β-catenin degradation) or ICG-001(works via binding to cyclic AMP response element-binding protein), the protective effect was attributed to increased epithelial differentiation of mesenchymal stem cells^47, 48^. In our CLP model iCRT3 treatment not only attenuated lung collagen deposition but also decreased the expression of proinflammatory cytokines IL-6, TNF-α, and IL-1β and chemokines MIP-2 and KC. MIP-2 and KC are reported to be sufficient to induce neutrophil recruitment to the lung^49^. Indeed, iCRT3 treatment also reduced excessive infiltration of neutrophils observed as MPO activity in the lungs of septic mice.

Apoptosis of immune and epithelial cells is an important mechanism contributing to acute lung injury and associated inflammation^50, 51^. By using TUNEL assay, we demonstrated that CLP induced significant apoptosis in the lungs of mice and iCRT3 treatment effectively decreased the number of apoptotic cells in the lungs of septic mice. Wnt/β-catenin signaling is known to regulate apoptosis through a variety of mechanisms, including TRAIL, caspases, STAT3, AKT, PTEN, PI3K, and MAPK pathways, enhancing or restraining it, depending upon cellular or environmental context^52^. Wnt/β-catenin-induced cell apoptosis has been reported in melanoma^53, 54^, and hepatocellular carcinoma^55^. In addition, activated Wnt/β-catenin signaling was shown to promote macrophage apoptosis in response to mycobacterial infection via caspase-3 dependent pathway^56^. Apoptosis of macrophages has been implicated in the pathogenesis of sepsis^57^. This supports our study as blocking Wnt/β-catenin signaling resulted in reduced apoptosis.

In order to test the effectiveness of iCRT3 at the hyper-inflammatory stage in sepsis, we administered iCRT3 at 5 h after CLP when the levels of most proinflammatory cytokines are markedly elevated in mice. This study is the proof-of-concept to show the potential of using iCRT3 against sepsis. As for the treatment window, dose, and frequency of iCRT3 administration as well as its toxicity and pharmacokinetics, all these require a series of pre-clinical studies to develop iCRT3 as a drug candidate for treating sepsis. To limit the interference from other treatments, antibiotic administration to these animals was avoided for this mechanistic study. Also, to reduce the variability in statistic analyses, only male mice were used in this study. To conduct any future pre-clinical studies to evaluate the efficacy of iCRT3, based on the positive outcomes observed in this study, the antibiotic administration and mixed gender issues also need to be considered to mimic the clinical setting. In this study, we have demonstrated the effectiveness of iCRT3 treatment on the reduction of inflammation, apoptosis, and lung injury in short-term. Whether its effect can extend to long-term benefit needs to be further determined in a survival study.

In conclusion, data provided in this study identifies that iCRT3 blocks the Wnt/β-catenin activity in macrophages to inhibit cytokine production and NFκB signaling. Treatment with iCRT3 significantly attenuates the sepsis-induced organ injury and systemic inflammation. In particular iCRT3 improves the histopathology of lung tissue and decreases lung collagen deposition. iCRT3 does so by effectively inhibiting the sepsis-induced excessive cytokine production, apoptosis and neutrophil infiltration in the lungs. Thus, Wnt/β-catenin signaling may be a potential therapeutic agent for sepsis.

## Methods

### Cell Culture

Mouse macrophage cell line RAW264.7 was purchased from ATCC (Manassas, VA). RAW264.7 cells were cultured in DMEM medium (Life Technologies, Grand Island, NY) containing 10% fetal bovine serum (FBS), 2 mM L-glutamine and 1% penicillin/streptomycin in a 37 °C incubator with 5% CO_2_.

### β-catenin-TCF reporter activity assay

RAW264.7 cells were seeded the day before transfection at a density of 1.24 × 10^5^ cells per ml. Cells were transiently co-transfected with 250 ng of TOP-TK-Luc or FOP-TK-Luc (Upstate Biotechnology, Lake Placid, NY) and 25 ng pRL-TK (Promega, Madison, WI) reporter plasmids, using the Lipofectamine 3000 Reagent (Thermo Fisher Scientific, Waltham, MA) according to the manufacturer’s instructions. At 24 h after transfection, cells were pre-treated with iCRT3 (EMD Millipore, Billerica, MA) or vehicle for 50 min and then stimulated with LPS (1 ng/ml) for another 24 h. The cells were lysed 48 h post-transfection and luciferase activity was measured with a Dual-Luciferase reporter assay system (Promega) according to the manufacturer’s instructions. TOP-TK-Luc contains optimal and FOP-TK-Luc contains mutated TCF-binding sites placed upstream of a firefly luciferase reporter gene. The TOP and FOP firefly luciferase activity was normalized to *Renilla* luciferase activity from the cotransfected pRL-TK plasmid used as an internal control for transfection efficiency. All experiments were performed in triplicate at least twice.

### Cell viability assay

Cell viability in each well was determined using a cell proliferation assay kit according to the manufacturer’s instruction (Promega, Madison, WI). Briefly, 20 μl of the assay reagent were added to each well of the 96 well plate containing 100 μl of cells in culture medium and incubated at 37 °C for 1–4 h in a humidified 5% CO2 atmosphere. The absorbance was recorded at 490 nm.

### Animal model of cecal ligation and puncture (CLP)-induced sepsis

Male C57BL/6 mice (20 to 25 g) purchased from Taconic Biosciences (Albany, NY) were used in all experiments at 8–12 weeks age. These mice were housed in a temperature-controlled room on a 12 h light/dark cycle in the animal facility within the Feinstein Institute for Medical Research (Manhasset, NY) to acclimate to the environment for at least 5 days before being used for experiments and fed a standard laboratory diet. All experiments were performed in accordance with the recommendations in the Guide for the Care and Use of Laboratory Animals of the National Institutes of Health (Bethesda, MD) and were approved by the Institutional Animal Care and Use Committee (IACUC) at the Feinstein Institute for Medical Research. All efforts were made to minimize suffering. Sepsis was induced in mice using CLP procedure. Briefly, the mice were anesthetized by isoflurane inhalation, and the abdomen was shaved and cleaned with 10% povidone iodine before operation. A 2-cm midline laparotomy was performed to expose the cecum. The cecum was tightly ligated (1 cm from the cecum tip) with a 4–0 silk suture distal to the ileocecal valve, double punctured with a 22-gauge needle, gently squeezed to expel small amount of feces and returned to the peritoneal cavity. The laparotomy site was then closed with a 6–0 silk suture in two layers and the animals were immediately resuscitated with 1 ml of normal saline injected subcutaneously. The sham animals underwent the same procedure but the cecum was neither ligated nor punctured. At 20 h after CLP or sham operation, mice were anesthetized and blood, lungs were collected. Blood samples were centrifuged to collect plasma and a section of lung tissue was preserved in formalin for histopathological analysis. The rest of lung tissues were immediately frozen in liquid nitrogen, and all the samples were stored at −80 °C until analysis.

### Administration of iCRT3

Mice were randomly allocated to three groups: sham (n = 5 mice), vehicle and treatment (n = 8 mice per group). iCRT3 (EMD Millipore, Billerica, MA) was reconstituted with cell culture grade 100% DMSO as 50 mg/ml stock. 5 and 10 mg/kg body weight (BW) concentrations of iCRT3 were made by diluting stock in sterile normal saline with 5% DMSO. At 5 h after CLP, 5% DMSO in normal saline (vehicle) or iCRT3 at 5 or 10 mg/kg BW doses in 200 μl volume was delivered by intraperitoneal injection using 25 G × 7/8″ hypodermic needle (Becton, Dickinson & Company, Franklin Lakes, NJ). The investigator performing the animal experiments was blinded to the treatment assignment to eliminate any bias.

### Measurements of cytokines and organ injury markers

TNF-α levels in the supernatants from RAW264.7 cultures and IL-6, TNF-α, and IL-1β levels in the plasma samples were quantified by using the specific mouse enzyme-linked immunosorbent assay (ELISA) kits (BD Biosciences, Franklin Lakes, NJ, USA). Plasma levels of aspartate aminotransferase (AST), alanine aminotransferase (ALT) and lactate dehydrogenase (LDH) were measured by using the commercial assay kits (Pointe Scientific, Lincoln Park, MI, USA) according to the manufacturer’s instructions.

### Histologic examination

The lung tissues were fixed in 10% formalin, paraffin embedded, cut into 5 μm sections, transferred to glass slides and stained with hematoxylin and eosin (H&E) and Masson’s-Trichrome. Morphologic changes in the lung tissues were examined under a light microscope, and evaluated by two independent investigators blinded to the treatment assignment. Lung injury was assessed according to the following pathological features: (i) alveolar mambrane thickening, (ii) vascular congestion, (iii) intra-alveolar hemorrhage, and (iv) interstitial and alveolar neutrophil infiltration. The semi-quantitative scores from 0 to 3 were designated based on absence or presence and severity of each of these features ranging from mild, moderate to severe and a cumulative total histology score was determined.

### Terminal deoxynucleotidyl transferase dUTP Nick End-Labeling (TUNEL) Assay

Lung tissue sections were deparaffinized, rehydrated, treated with Proteinase K and stained with TUNEL staining kit (Roche Diagnostics, Indianapolis, IN) according to the manufacturer’s instructions to detect the presence of apoptotic cells. The negative control was performed by incubating slides in the mixture containing only deoxynucleotidyl transferase. TUNEL-positive cells were counted under a fluorescence microscope across 10 microscopic fields per section at 200 × magnification.

### Western blotting analysis

RAW264.7 cells were homogenized in lysis buffer (10 mM Tris-HCl, pH 7.5, 120 mM NaCl, 1% NP-40, 1% sodium deoxycholate, and 0.1% SDS) containing a protease inhibitor cocktail (Roche Diagnostics, Indianapolis, IN) by sonication. Protein concentrations were determined by *DC* protein assay (Bio-Rad Laboratories, Hercules, CA). Total cell lysates were fractionated on Bis-Tris gels (4 to 12%) and transferred to nitrocellulose membrane. The membranes were then blocked with 0.1% casein (Sigma-Aldrich, St Louis, MO, USA) in phosphate-buffered saline and probed with anti-IκB (Santa Cruz Biotechnology, Santa Cruz, CA) or anti-β-actin (Sigma-Aldrich, St Louis, MO) antibodies. After the wash, the membranes were incubated with the appropriate fluorescence-labeled secondary antibodies (LI-COR Biosciences, Lincoln, NE) and scanned by the LI-COR Odyssey Fc Imager (LI-COR Biosciences).

### Quantitative PCR (qPCR) analysis

TRIzol (Thermo Fisher Scientific, Waltham, MA) was used to extract total RNA from the lung tissue homogenates. RNA was reverse-transcribed into cDNA using murine leukemia virus reverse transcriptase (Thermo Fisher Scientific, Waltham, MA). A PCR reaction was carried out in 20 μl of a final volume containing 0.06 μM of each forward and reverse primer, cDNA, and 10 μl SYBR Green PCR Master Mix (Applied Biosystems, Foster City, CA). Amplification was conducted in an Applied Biosystems StepOnePlus real-time PCR machine under the thermal profile of 50 °C for 2 min, 95 °C for 10 min followed by 45 cycles of 95 °C for 15 sec and 60 °C for 1 min. For relative quantification, ΔΔCT comparative threshold cycle (C_T_) method, normalized to mouse β-actin mRNA was used. Relative expression of mRNA was expressed as the fold change compared to the sham. The primers used for this study are listed in Table 1.

**Table 1:** Sequences of the primers used in qPCR.

Gene	Forward primer sequence	Reverse primer sequence
IL-6	CCGGAGAGGAGACTTCACAG	GGAAATTGGGGTAGGAAGGA
TNF-α	AGACCCTCACACTCAGATCATCTTC	TTG CTACGACGTGGGCTACA
IL-1β	CAGGATGAGGACATGAGCACC	CTCTGCAGACTCAAACTCCAC
MIP-2	CCCTGGTTCAGAAAATCATCCA	GCTCCTCCTTTCCAGGTCAGT
KC	GCTGGGATTCACCTCAAGAA	ACAGGTGCCATCAGAGCAGT
β-actin	CGTGAAAAGATGACCCAGATCA	TGGTACGACCAGAGGCATACAG

### Myeloperoxidase (MPO) activity assay

Lung tissues were homogenized in potassium phosphate buffer containing 0.5% hexa-decyl-trimethyl-ammonium bromide by sonication. After centrifugation the supernatant was diluted in reaction solution containing o-dianisidine hydrochloride and hydrogen peroxide. The rate of change in optical density per minute was measured at 460 nm to calculate MPO activity.

### Statistical analysis

Data were analyzed using SigmaPlot11 graphing and statistical analysis software (Systat Software Inc., San Jose, CA) and expressed as mean ± standard error of the mean (SEM). Multiple groups were compared with one-way analysis of variance (ANOVA) using Student-Newman-Keuls’ (SNK) test. Differences in values were considered significant if *P* < 0.05.

### Data Availability

All data generated or analyzed during this study are included in this published article.
